The article "Evaluation of the Anticancer Potential of Morus nigra and Ocimum basilicum Mixture against Different Cancer Cell Lines: An In Vitro Evaluation" was retracted in 2024. Reasons: signs of a paper mill; suspected computer-generated content; unreliable results or conclusions; concerns about the data.

# Evaluation of the Anticancer Potential of *Morus nigra* and *Ocimum basilicum* Mixture against Different Cancer Cell Lines: An In Vitro Evaluation

**DOI:** 10.1155/2023/9337763

**Published:** 2023-04-19

**Authors:** Bader O. Almutairi, Ahmed I. Alsayadi, Nael Abutaha, Fahd A. AL-mekhlafi, Mohamed A. Wadaan

**Affiliations:** Department of Zoology, College of Science, King Saud University, P.O. Box 2455 Riyadh 11451, Saudi Arabia

## Abstract

*Morus nigra* (M) and *Ocimum basilicum* (O) mixture (MO2) extract was extracted using hexane (MO2H), chloroform (MO2C), ethyl acetate (MO2E), and methanol (MO2M) in a Soxhlet apparatus. The cytotoxicity was evaluated using MTT (3-[4,5-dimethylthiazol-2-yl]-2,5 diphenyl tetrazolium bromide) assay. The IC_50_ values of the MO2C-treated cancer cells were 11.31 *μ*g/mL (MDA-MB-231), 15.45 *μ*g/mL (MCF-7), 18.9 *μ*g/mL (HepG2), 26.33 *μ*g/mL (Huh-7), 30.17 *μ*g/mL (LoVo), and 36.76 *μ*g/mL (HCT116). MO2C-treated cells showed cellular and nuclear morphological alterations like chromatin condensation and formation of apoptotic bodies as observed using light and fluorescent microscopy. The antioxidant and anti-inflammatory properties were investigated in vitro using 2,2′-diphenyl-1-picrylhydrazyl (DPPH) and egg albumin denaturation assays. It was evident that the MO2M extract exhibited the highest antioxidant activity (18.13%), followed by the MO2E extract (12.25%), MO2C extract (9.380%), and MO2H extract (6.31%). The highest inhibition percentage of albumin denaturation was observed in MO2H (28.54%), followed by MO2M (4.32%) at 0.2 and 0.1 mg/mL concentrations, respectively. The compounds identified using gas chromatography-mass spectrometry (GC-MS) analysis for MO2C extract were *α*-trans-bergamotene, germacrene D, selin-4,7(11)-diene, 2 tridecen-1-ol, and 2-decen-1-ol. The present study reveals that MO2C has promising anticancer activity and may serve as a potent polyherbal extract in cancer treatment.

## 1. Introduction

There is an increase in the incidence of cancer and death cases worldwide [1], and this could be attributed to lifestyle changes (tobacco smoking, alcohol, diet, and obesity) and environmental factors (air and water pollution) [2]. In Saudi Arabia, the estimated numbers of new cancer cases and deaths in 2020 are 27885 and 13069, respectively. Among distinct types of cancer, breast cancer is considered the leading cause of mortality and morbidity in females living in Saudi, with approximately 1095 deaths. In Saudi Arabia, the most frequently recorded cancer cases in males and females are colorectal and breast cancers, respectively. In females, breast cancer constitutes 29% of the confirmed cancer cases, followed by thyroid (14.3%) and colorectal (9.2%) cancer. In contrast, colorectal cancer represents 19.3%, non-Hodgkin lymphoma 8%, leukemia 6.7%, and thyroid 6.2% of the total reported cases in males [3].

Surgery, chemotherapy, radiation therapy, proton therapy, and immunotherapy are cancer treatment methods that have been commonly used to treat cancer [4]. Unfortunately, these approaches can induce adverse effects on patients, causing them more discomfort. Sometimes, they are not sufficiently effective. Moreover, cells may develop resistance even to recently synthesized drugs. Despite the positive effects that pharmaceutical anticancer drugs may exert, such drugs may also cause harmful reactions, including hypertension, lung damage, menopausal symptoms, change in sexual desire, osteoporosis, cardiotoxicity, brain and spinal cord problems, nerve disorders, and hair loss accompanied by vomiting [5]. Therefore, more studies are being conducted to explore new and safe anticancer agents from botanical sources that can prevent or suppress carcinogenesis [6, 7].

The life expectancy of cancerous cells is greatly affected by the rate of apoptosis. Therefore, modulating apoptosis may probably be helpful towards cancer treatment and prevention. In fact, natural products can markedly induce apoptotic mechanisms [8, 9]. The cytotoxic and apoptotic activities of polyherbal extracts were previously reported. An extract which was developed by mixing the root extract of *Hemidesmus indicus* (roots), *Nigella sativa* (seeds), and *Smilax glabra* rhizomes together exerted high cytotoxicity against NCI-H292 (lung cancer cells) and weaker cytotoxic effects on MRC-5 (normal lung cells) [10]. Similarly, a polyherbal medicine, “Le Pana Guliya” showed antiproliferative effects against HeLa and HepG2 cells with an IC_50_ value of 19.03 and 2.72 *μ*g/mL, respectively. The Le Pana Guliya extract exerted anticancer effects through oxidative stress-dependent apoptosis [11]. Accordingly, this study evaluated the cytotoxicity and apoptotic potential of *Morus nigra* (black mulberry) and *Ocimum basilicum* (sweet basil) mixture against different cancer cell lines.

## 2. Research Methodology

### 2.1. Selection of Plants

Dried leaves of *Morus nigra* L. and *Ocimum basilicum* L. were purchased from a herbal store called Bin Menqash, located on Imam Saud Bin Abdulaziz Road, Riyadh, Saudi Arabia. The dried herbs were examined and identified by a taxonomist at the Botany and Microbiology Department at King Saud University.

### 2.2. Preparation of Polyherbal Extracts

The polyherbal extracts were prepared by mixing equal quantities of *M. nigra* (20 g) and *O. basilicum* (20 g). Then, the herbs were grinded by a coffee grinder. Subsequently, their powder was extracted via Soxhlet extractor using four solvents (450 mL each) of different polarities. The employed solvents were hexane, chloroform, ethyl acetate, and methanol (Sigma-Aldrich, France), respectively. Next, the four polyherbal extracts were evaporated using a rotary evaporator (Heidolph, Germany) at 45°C. Then, they were dissolved in DMSO (Panreac, E.U) and transferred into small tubes. Eventually, the tubes were labeled and preserved at -20°C.

### 2.3. Total Polyphenol Content

The total phenol content was evaluated through the Folin-Ciocalteu (Alpha Chemika, India) assay method [12]. Two microliters of each extract was mixed with twenty microliters of Folin-Ciocalteu reagent (10%) in a 96-well plate. Then, the mixture was triturated a few times and kept for ten minutes at 25°C. Subsequently, 80 *μ*L of 7.5% sodium carbonate was pipetted into the wells and mixed for a couple of times. Then, the 96-well plate was incubated at 25°C for two hours to observe any color change. Lastly, the wells' absorbances were measured at 765 nm using a microplate reader (ChromMate, UK). The total phenolic content was recorded as mg/g gallic acid (GAE/g) equivalent according to the standard curve (*y* = 0.0042 × +0.0489, *R*^2^ = 0.97).

### 2.4. Total Flavonoid Content

The total flavonoid content was evaluated using the aluminium chloride (AlCl_3_) colorimetric assay [12]. In a 96-well plate, 2 *μ*L of each plant extract was combined with 60 *μ*L of methanol, of 10% aluminium chloride (4 *μ*L), 1 M of potassium acetate (4 *μ*L), and 112 *μ*L of distilled water. After that, the mixture was triturated for a few seconds and then incubated for 30 minutes. Thereafter, the mixture was read at 420 nm via a spectrophotometer. The total flavonoid content was documented as mg/g quercetin equivalent according to the standard curve (*y* = 0.0032 × +0.0492, *R*^2^ = 0.99).

### 2.5. Gas Chromatography-Mass Spectrometry (GC-MS)

As carried out earlier, the compounds found in MO2C extract were investigated using GC-MS (Agilent Technologies, USA) [13]. Those phytochemicals were identified by comparing their mass spectra to the library of the National Institute of Standards and Technology (NIST, 2004).

### 2.6. DPPH Radical Scavenging Assay

The radical scavenging activity of the MO2 extracts was evaluated *in vitro* following the method instructed by Abutaha et al. [12]. The reaction solution composed of 198 *μ*L DPPH (0.008% in methanol) and 2 *μ*L of various extract concentrations (4–0.125 mg/mL) of each plant, as well as standardizing gallic acid (10–90 *μ*g/mL). The components were mixed in a 96-well plate and kept in the dark at 25°C for half an hour. Subsequently, the absorbances of the wells were measured at 517 nm using a plate reader. In addition, the percentage of the DPPH radical scavenging activity was calculated based on the standard curve.

### 2.7. Cell Culture

Double negative MDA-MB-231^ER(−)/PR(−)^, double-positive MCF-7 ^ER(+)/PR(+)^ estrogen receptor (ER) and progesterone receptor (PR) human breast adenocarcinoma cell lines, human hepatoma (HepG2, Huh-7, and CHANG), human colorectal carcinoma (HCT116 and LoVo), and human umbilical vein endothelial cells (HUVEC) were obtained from the Leibniz-Institute DSMZ-German Collection of Microorganisms and Cell Cultures and Japanese Tissue Culture. The cells were cultured in Dulbecco's Modified Eagle Medium (DMEM) (Gibco, USA) supplemented with penicillin (100 U/mL) and streptomycin (100 *μ*g/mL) (Gibco, USA) and 10% fetal bovine serum (Gibco, USA). Cells were grown at 37°C in a CO_2_ incubator (5% CO_2_) and using trypsin-EDTA solution (Gibco, USA).

### 2.8. Cytotoxicity Assays

Through the MTT assay, the extracts were assessed for their cytotoxic effects on eight cell lines. In 24-well plates, the cells were plated at 10^5^ cells/mL density in Dulbecco's Modified Eagle Medium (DMEM) with 10% fetal bovine serum at 37°C in 5% CO_2_ [14]. Additionally, the plates were kept in the incubator for 24 hours. Then, they were treated using various concentrations of the plant extracts for another 24 hours. In addition, DMSO-treated (0.5%) wells served as negative controls, and carbonyl cyanide 3-chlorophenylhydrazone was used as a positive control. After the 24-hour treatment, the MTT solution was pipetted into the wells and incubated for 2 hours. Subsequently, the formazan crystals were dissolved using a solubilization solution such as DMSO. The resulting-colored solution was quantified by reading the absorbances of samples at 570 nm via a spectrophotometer [12].

### 2.9. Morphological Changes by Light Microscopy

Cells were exposed to MO2C extract for 24 h. After the treatment period, cells were observed under light microscope (Leica, Germany) to detect apoptosis morphological changes.

### 2.10. DAPI (4′,6-Diamidino-2-phenylindole) Staining

Initially, cells were cultured and then treated at a proper confluence (70%). Phosphate-buffered saline (1X PBS, pH 7.4) was applied to wash the treated cells. Then, the cells were fixed in 70% ethanol for five minutes. After that, they were stained with DAPI dissolved in PBS (5 *μ*L/mL) and incubated for half an hour at 37°C in the dark. Next, the cells were washed using PBS and examined by fluorescent microscopy.

### 2.11. In Vitro Anti-inflammatory Bioassay

The protein denaturation assay was carried out based on the method demonstrated by [15]. Five millilitres of the reaction mixture (0.02 mL of extract, 4.78 mL of PBS (pH 6.4), and 0.2 mL of 1% bovine albumin) was incubated for fifteen minutes at 37°C and subsequently heated at 70°C for 5 minutes. Upon cooling, the turbidity was assessed at 660 nm by a plate reader. Also, PBS solution was employed as a control. The percentage inhibition of protein denaturation was found by using the following equation:

%inhibition = 100 × [Vt/Vc–1]; Vt represents the absorbance of the test sample, whereas Vc refers to the absorbance of the control.

## 3. Result

### 3.1. Phenolic and Flavonoid Contents of Tested Extracts

The total phenolic content was found to be at its highest level in the ethyl acetate extract (36.69 mg gallic acid equivalent (GAE)/g dry weight), followed by methanol (33.23 mg GAE/g dry weight), chloroform (11.61 mg GAE/g dry weight), and hexane (7.510 mg GAE/g dry weight) extract. Moreover, the total flavonoid content results showed that the ethyl acetate extract had the maximum value (22.95 mg quercetin equivalent (QE)/g dry weight) followed by chloroform (7.75 mg QE/g dry weight), methanol (6.75 mg QE/g dry weight), and hexane (6.47 mg QE/g dry weight) extract.

### 3.2. Composition Analysis of the Extract

The chromatogram and the identified compounds are presented in Table 1 and Figure 1. A total of 5 phyto-compounds were identified in the MO2C extract. The compounds identified were *α*-trans-bergamotene, germacrene D, selin-4,7(11)-diene, 2-tridecen-1-ol, and 2-decen-1-ol.

### 3.3. In Vitro Antioxidant Activity

The *in vitro* antioxidant activity assays were performed to evaluate the capacity of herbal extracts to scavenge free radicals DPPH. Overall, it was apparent that MO2M possessed the highest antioxidant properties (18.13%), followed by MO2E (12.25%), MO2C (9.380%), and MO2H (6.31%) (Table 2).

### 3.4. In Vitro Anti-inflammatory Bioassay

The anti-inflammatory properties of MO2 extracts were assessed using the egg albumin method. The highest inhibition percentage was observed in MO2H (28.54%) followed by MO2M (4.32%) at 0.2 and 0.1 mg/mL concentrations, respectively.

### 3.5. Cytotoxic Effects

A normal cell line and seven distinct cancer cell lines were incubated with different concentrations of solvent extracts for 24 hours to determine the effectiveness of each extract based on their corresponding cytotoxic effects. The results indicated that only the chloroform extract (MO2C) was toxic against all cell lines but CHANG cells at the highest concentration. (Figures 2 and 3). The IC_50_ values of the MO2C-treated cancer cells were 11.31 *μ*g/mL (MDA-MB-231^ER(-)/PR(-)^), 15.45 *μ*g/mL (MCF-7^ER(+)/PR(+)^) 18.9 *μ*g/mL (HepG2), 26.33 *μ*g/mL (Huh-7), 30.17 *μ*g/mL (LoVo), and 36.76 *μ*g/mL (HCT116). MDA-MB-231^ER(−)/PR(−)^ cells were the most sensitive cancer cell line tested with an IC_50_ value of 11.31 *μ*g/mL. In addition, HCT116 cells were the least sensitive with an IC_50_ value of 36.76 *μ*g/mL. MO2C extract displayed selective cytotoxicity because it was less toxic to the normal HUVEC cells (IC_50_: 38.45) compared to the other cancer cell lines. Carbonyl cyanide 3-chlorophenylhydrazone was used as a positive control, and its calculated IC_50_ values were 1.36, 2.26, 10.67, 18.39, 29.06, 53.27, and 44.98 *μ*g/mL against Huh-7, MDA-MB-231, HCT116, MCF7, LoVo, HepG2, and HUVEC cells, respectively.

### 3.6. Cell Morphology and DAPI Staining

The morphology of the MCF-7 cells was affected by MO2C extract, whereas the control cells showed typical cell morphologies. Shrinkage, cell detachment, complete cellular integrity loss, and cytoplasm contraction were observed in MCF-7 cells treated with MO2C extract (Figure 4). The effect of MO2C extract on the nuclear morphology of MCF-7 cells was assessed by DAPI staining. As exhibited in Figure 4, MO2C extract-treated cells showed chromatin condensation and formation of apoptotic bodies. In contrast, the control cells were stained uniformly (Figure 4) and morphologically intact. They were adherent to the surface and tightly packed.

## 4. Discussion

According to the United States National Cancer Institute plant screening program, the cytotoxic activity of crude extracts is promising if the IC_50_ value is <30 *μ*g/mL [16]. The MO2C extract was cytotoxic at very low concentrations. Its cytotoxic activity against HepG2, MCF-7, HCT116, LoVo, MDA-MB-231, and Huh-7 was selective compared to the normal human umbilical vein endothelial cells (HUVECs). To date, most chemotherapeutic agents attack both normal and cancer cells indiscriminately. For less damage to normal cells postcancer therapy, it is essential to develop natural product extracts with selective cytotoxicity towards cancer cells. Thus, plant extracts cytotoxic effects on cancer cells were compared to that of normal HUVEC cells. Different researchers observed similar results such as the selective cytotoxicity observed in *Artemisia absinthium* leaf and seed extract on A-549, K-562, K-562, MCF-7, and PC-3 cells compared with human bronchial epithelial cell line (BEAS-2B) [17]. Similarly, researchers claimed that the *Primula auriculata* and *Primula vulgaris* extract exhibited selective cytotoxic effects on different human cancer cell lines, including MCF-7, HepG2, HT-29, A549, PC-3, and WiDr compared with normal bovine kidney cells and human normal fibroblast cells [18, 19].

It is noted that different cancer cell lines may respond to cancer drugs differently [20, 21]. In this study, it was noticeable that there were variations in response to MO2C extract from different cell lines derived from the same organs, such as breast cancer MCF7 and MDA-MB-231, colon cancer HCT116, LoVo, and liver cancer HepG2, Huh-7, and CHANG. It has been widely acknowledged that many tumors are not homogenous in nature but are comprised of cells of different characteristics. Tumoral heterogeneity occurs in many cancers causing different resistances to treatment, drug sensitivities, and relapse after treatment [22, 23]. Therefore, tumor heterogeneity is a significant obstacle in cancer treatment. Hence, cellular heterogeneity is an important factor in assessing the overall response of cells to cancer drug treatment. Therefore, drug combination and botanical extract serve as promising resources towards the mission of overcoming this obstacle.

Plant extracts are a valuable source of anticancer agents [24]. Secondary metabolites such as polyphenols, flavonoids, terpenoids, and alkaloids exhibit different biological activities, such as antioxidant, anti-inflammatory, anticancer, and antiaging [25]. In fact, several polyphenols and flavonoids have already been reported for their anticancer activities such as hydroxycinnamates, lignins, chalcones, stilbenes, xanthones, coumarins, flavonoids, and hydroxybenzoates [26].

Anticancer agents that induce apoptosis are considered as one of the most effective strategies of chemotherapy [27]. Thus, when searching for new anticancer agents, the candidates should demonstrate apoptosis induction in cancer cells [28]. Our data showed that MO2C treatment resulted in the formation of apoptotic bodies, membrane blebbing, cell shrinkage, and other morphological changes, all of which are common features of apoptosis [29, 30]. Upon application of DAPI staining, the treated cells displayed chromatin condensation and nuclear fragmentation, which could be associated with apoptosis induction relative to normal control cells (Figure 4). Similar results have been published where polyherbal extracts showed apoptotic activity against MCF-7 and other cancer cells [31–33].

Protein denaturation causes the production of auto-antigens in different medical conditions such as diabetes, rheumatic arthritis, and cancer, which are recognized as chronic inflammatory disorders. Therefore, by inhibiting protein denaturation, inflammation is also inhibited [34]. The egg albumin method provides a cheap alternative way of testing the anti-inflammatory activity of herbal medicines. In the future, the anti-inflammatory test of MO2C should be validated by in vivo and in vitro studies such as rat paw edema, bovine serum albumin, and membrane stabilization. From phytochemical investigation, the presence of different compounds suggested that one of the constituents or their combination is responsible for producing the anti-inflammatory effects.

The compounds identified by GC-MS in the present sample (Table 1 and Figure 1), namely, germacrene D, *α*-*trans*-bergamotene, selin-4,7(11)-diene, 2-decen-1-ol, and 2-tridecen-1-ol were not individually tested. Still, they have been associated with the anticancer and anti-inflammatory activities of many plants' crude extracts [35–40]. In addition, in silico molecular docking conducted by Farooq Khan et al. showed that the possible molecular mechanism of anticancer activity is the binding of 2-Tridecen-1-ol with phase inducer phosphatases 2 with higher binding energy as compared to M-phase inducer phosphatases [37].

## 5. Conclusion

This study demonstrates the anticancer potential of *M. nigra* and *O. basilicum* mixture for the first time against different cancer cell lines. Further studies on combining the extract with other anticancer drugs and in vivo animal models are necessary before advancement to clinical trials.

## Figures and Tables

**Figure 1:** Gas chromatography-mass spectrometry chromatogram of MO2C.

**Figure 2:** Dose-dependent cytotoxic effect of MO2C extract and cyanide 3-chlorophenylhydrazone after 24 hours of exposure on human cancer cell lines, namely, hepatocellular carcinoma (HepG2, CHANG), human colon carcinoma (HCT116), and the normal human umbilical vein endothelial cells (HUVECs).

**Figure 3:** Dose-dependent cytotoxic effect of MO2C extract and cyanide 3-chlorophenylhydrazone after 24 hours of exposure on different human cancer cell lines, namely, hepatocellular carcinoma (Huh-7), human colon carcinoma (LoVo), and human breast carcinoma (MCF7 and MDA-MB-231).

**Figure 4:** Morphological and nuclear assessment of MO2H-treated and untreated cells MCF-7ER(+)/PR(+) cells at IC_50_ × 2 after 24 h. Cells were observed using light and fluorescent microscopes. (a) DMSO treated MCF-7ER(+)/PR(+) cells after 24 h. (b) Detachment of cell from culture plate (BT549) after 24 h exposure to MO2H at IC_50_ × 2 value. (c) Control cells stained with DAPI appear evenly stained with no DNA fragmentation. (d) MCF7 cells treated with MO2H extract show apoptotic nuclei. Images are magnified at 40×. Scale bars = 100 *μ*m.

**Table 1:** Phytochemical profile of MO2C extract using gas chromatography-mass spectrometry.

No.	Compounds	Retention time	Area %	Formula	Molecular weight
1	*α*-*Trans*-bergamotene	10.58	8.930	C_15_H_24_	204.35
2	Germacrene D	11.47	2.800	C_15_H_24_	204.35
3	Selin-4,7(11)-diene	12.69	19.620	C_15_H_24_	204.35
4	2-Decen-1-ol	14.13	62.820	C_10_H_20_O	156.26
5	2-Tridecen-1-ol	14.31	5.840	C_13_H_26_O	198.34

**Table 2:** Total polyphenols and total flavonoids contents, antioxidant, and anti-inflammatory activities of different solvent extract of *M. nigra* and *O. basilicum* mixture.

No.	Sample	Total flavonoid content (1 mg/mL)	Total polyphenol content (1 mg/mL)	Antioxidant DPPH (% inhibition at 4 mg con.)	Anti-inflammatory (% inhibition of albumin denaturation at 1 mg con. except MO2H at 0.5 mg)
1	MO2H	6.47	7.510	6.31	28.54
2	MO2C	7.75	11.61	9.38	—
3	MO2E	22.95	36.69	12.25	—
4	MO2M	6.75	33.23	18.13	4.32

## Data Availability

All the data relevant to this study is mentioned in the manuscript. There is no supplementary data.
